The article "Antiangiogenic Potential of Troxerutin and Chitosan Loaded Troxerutin on Chorioallantoic Membrane Model" was published in 2023. Journal: Biomed Res Int.

# Antiangiogenic Potential of Troxerutin and Chitosan Loaded Troxerutin on Chorioallantoic Membrane Model

**DOI:** 10.1155/2023/5956154

**Published:** 2023-05-23

**Authors:** Gowtham Kumar Subbaraj, Harini Elangovan, Prema Chandramouli, Santhosh Kumar Yasam, Kirubhanand Chandrasekaran, Langeswaran Kulanthaivel, Sangavi Pandi, Senthilkumar Subramanian

**Affiliations:** ^1^Faculty of Allied Health Sciences, Chettinad Hospital and Research Institute, Chettinad Academy of Research and Education (Deemed to be University), Kelambakkam, 603 103 Tamil Nadu, India; ^2^Department of Anatomy, All India Institute of Medical Sciences (AIIMS), Nagpur, Maharashtra, India; ^3^Cancer Genetics & Molecular Biology Laboratory, Department of Biotechnology, Science Campus, Alagappa University, Karaikudi, Tamil Nadu 630003, India; ^4^School of Medicine, College of Medicine and Health Science, Jigjiga University, Ethiopia

## Abstract

Angiogenesis is crucial to the development of cancer because it allows the transport of oxygen, nutrients, and growth factors as well as the spread of tumors to distant organs. Inhibitors of angiogenesis prevent the formation of blood vessels that allow tumor cells to shrink, rather than promote tumor growth. Chitosan acts as a carrier for many drugs, since the compound has various properties such as biodegradable, less toxicity, more stable, simple, easy to prepare, and biocompatible. The aim of the current study was to evaluate the efficacy of chitosan nanoparticles encapsulated with troxerutin (Chi-Trox NPs) against angiogenesis and cancer *in ova* chick chorioallantoic membrane (CAM) model. Chi-Trox NPs were synthesized using a nanoprecipitation method and were characterized by various analyses. 24 hours' fertilized eggs (6 eggs/group) were treated with native Trox and Chi-Trox NPs for 5 days. The antiangiogenic activity was evaluated by morphometric, histopathological, immunohistochemical (CD104 and vimentin), and mRNA expression of MMP and FGF2 using RT-PCR. The anticancer activity was evaluated by histopathological, immunohistochmical (CD44), and mRNA expression of FGF2 and MMP. The synthesized chitosan NPs were successfully encapsulated with troxerutin, and the loading efficiency of chitosan NPs was found to be 86.4 ± 0.12% and 13.2 ± 0.16% respectively. Morphometric analysis of Chi-Trox NPs showed a considerable decrease in the number of blood vessels compared with control and native Trox. The histopathological observation of CAM confirmed that Chi-Trox NPs induce a significant reduction in inflammatory cells and the thickness of blood capillaries compared to control and native Trox. The immunohistochemical evaluation of CAM revealed Chi-Trox decreased CD104, vimentin and CD44 protein levels were compared with control and native Trox. Furthermore, the mRNA expression levels of FGF2 and MMP were significantly downregulated compared to their native forms. From the obtained results, Chi-Trox NPs possess significant inhibition of angiogenesis and can be used as therapeutic agents for cancer in the future.

The article "Antiangiogenic Potential of Troxerutin and Chitosan Loaded Troxerutin on Chorioallantoic Membrane Model" was published in 2023. Journal: Biomed Res Int.

## 1. Introduction

Angiogenesis is the process by which new blood vessels are generated from preexisting vessels in the early stages of vasculogenesis [1]. The process of angiogenesis plays a critical role in cancer growth, as solid tumors require blood supply to grow. A tumor can actually cause angiogenesis by emitting chemical signals that stimulate it. The newly formed blood vessels take oxygen and nutrients, allowing the tumors to grow and invade, thereby enabling the cancerous cells to spread throughout the body [2]. Proangiogenic and antiangiogenic factors control the growth of new blood vessels. Fibroblast growth factor (FGF) and vascular endothelial growth factor (VEGF) are proangiogenesis agents, while endostatin and TGF are antiangiogenesis agents [3, 4]. Flavonoids are secondary plant compounds that are frequently present in fruits, vegetables, and certain drinks. Flavonoids are known to have a broad range of health promoting effects [5]. As of now, flavonoids and their subordinates have been studied for their effectiveness in inhibiting the growth of cancerous cells and regulating vascular growth [6]. A significant challenge to cancer management is the cost-effectiveness of the current treatments. This burden causes immense economic hardship for societies around the world. Thus, the use of natural substances such as flavonoids for the prevention as well as the treatment of cancer can be considered an alternative therapeutic strategy [7].

Troxerutin, commonly known as vitamin P4, is a derivative of the bioflavonoid rutin, which can be found in tea, coffee, cereal grains, and a variety of vegetables and fruits [8]. Because of its high water solubility, troxerutin has been found to be readily absorbed by the gastrointestinal system and to produce protective effects without being cytotoxic [9]. This naturally occurring troxerutin has a number of biological functions, such as fighting cancer, reducing inflammation, fighting free radicals, and fighting diabetes.

Chitosan is a type of polymer that provides excellent protection and may be utilized for the delivery of active substances [10]. The encapsulation of flavonoids with chitosan nanoparticles has only been briefly studied in the past [11–13]. Compared to bulk chitosan, chitosan nanoparticles are used more frequently in biological applications because of their physicochemical properties, which include size, surface area, cationic nature, active functional groups, high permeability towards biological membranes, nontoxicity to humans, cost-effectiveness, higher encapsulation efficiency and/or through blending with other components, and broad biological activities. Chitosan nanoparticles have been employed in the distribution of active components due to their capacity to provide protection and stability. They offer defense against oxidation and enzymatic degradation as well as breakdown or damage brought on by exposure to oxygen, light, heat, and pressure [14, 15]. In the past few years, the chick chorioallantoic membrane (CAM) assay has emerged as the best tumor model among others, which provides a suitable and powerful system to assess the ability of nanoparticles to deliver anticancer drugs [16]. The CAM is formed during the development of the avian allantois and chorion. In a short period of time, this structure expands, creating a rich vascular network that functions as an interface for gas and waste exchange [17]. The CAM assay is preferable over other *in vivo* or *in vitro* models because it is highly sensitive and cost-effective. The aim of the present study was to prepare and characterize chitosan nanoparticles encapsulated with troxerutin and examine their antiangiogenic and anticancer efficacy in a CAM model.

The article "Antiangiogenic Potential of Troxerutin and Chitosan Loaded Troxerutin on Chorioallantoic Membrane Model" was published in 2023. Journal: Biomed Res Int.

## 2. Materials and Methods

Troxerutin (CAS-7085-55-4) was purchased from Cayman chemicals, USA. Chitosan (CAS-448869) was purchased from Sigma Aldrich, USA. Ethanol (64-17-5) was purchased from Changshu Chemicals Co., Ltd., China. Fertilized eggs were purchased from Tamil Nadu Veterinary and Animal Sciences University, Chennai, India. Anti-vimentin (SKU: AM074GP), CD34 (AN779GP) antibodies were purchased from BioGeneX, USA. Primers used were as follows: FGF2 (Forward: 5′CCTGGCACTGAATGTGCAAC3′; Reverse: 5′AACCCTCATTAAAGGGCAGACA3′) and MMP (Forward: 5′GTTACCACAGCGGGGTTTCT3′; Reverse: 5′TTTCAGATGGAAAACCAAGATGGA3′); c-DNA synthesis kit (6110A) were purchased from Takara, USA. TRIzol reagent (15596026) was obtained from Invitrogen, USA. All other compounds employed in the experiment were of an analytical grade.

### 2.1. Docking Studies

#### 2.1.1. Sequences and Homologous Analysis

The amino acid sequences are extracted from the primary database UniProt. To identify the homologous structure of the protein BlastP search was performed against the protein data bank [18]. From this search, evolutionary and functional relationships between protein sequences were analyzed.

#### 2.1.2. Exploration of Physicochemical Properties

Physicochemical properties were analyzed using the ProtParam tool [19]. This tool computationally predicts the total number of amino acids, molecular weight, iso-electric point, gravy, negatively charged amino acid, and positively charged amino acid present in the protein.

The article "Antiangiogenic Potential of Troxerutin and Chitosan Loaded Troxerutin on Chorioallantoic Membrane Model" was published in 2023. Journal: Biomed Res Int.

#### 2.1.3. Protein Structure Modeling

From the blast result, protein structure will be predicted by homology modeling or template-based modeling. High identity and query coverage lead to homology modeling. Homology modeling was constructed using the prime module in Schrodinger (Prime, Schrodinger, LLC, New York, NY, USA, 2021). Low identity and query coverage protein lead to template-based protein structure prediction. Template-based protein modeled using LOMETS server [20]. A three-dimensional protein structure was refined using galaxy web [21].

#### 2.1.4. Protein Structural Validation

Three-dimensional modeled protein validated in SAVES server. The stereo chemical property of the targeted protein was analyzed using PROCHECK tool [22]. The quality of protein was checked in the Ramachandran plot. The Ramachandran plot helps to determine the quality of protein using amino acid present in the protein structure. The Ramachandran plot favored region was represented by red color. Additional allowed region was represented by yellow color. White region in the plot shows the disallowed region present in the protein structure.

#### 2.1.5. Target Preparation and Ligand Preparation

Targeted protein was prepared in the protein preparation wizard in Schrodinger software (Impact, Schrodinger, LLC, New York, NY, USA, 2021). Targeted protein was prepared for further studies. Protein preparation includes removal of water molecules from the structure, add hydrogen atoms, and optimize the hydrogen bond using PROPKA minimization. This step helps to remove atomic clashes. During protein preparation protein structure was simulated using OPLS_2005 force field. The potential ligand molecules were in the LigPrep tool. LigPrep tool was embedded in the Schrodinger software (LigPrep, Schrodinger, LLC, New York, NY, USA, 2021). This tool helps to generate the accurate ligand with its appropriate ionization states and energy ring conformation. LigPrep OPLS_2005 force field was used to generate ligand molecules. Using LigPrep, we can remove improper ligand molecules.

#### 2.1.6. Active Site and Receptor Grid Generation

An active site is essential for inhibitor action of small molecules. A ligand molecule binds in the active site of the protein. The active site pocket of the protein was predicted by sitemap module present in the Schrodinger module (SiteMap, Schrodinger, LLC, New York, NY, USA, 2021). The active site was predicted based on the physical descriptor of the protein such as site volume and size of the site. A sitemap helps to identify the best using site score. Receptor grid generation using the glide module in Schrodinger (Receptor Grid Generation, Schrodinger, LLC, New York, NY, USA, 2021). Receptor grid generation plays a vital role in validation of specific receptor molecules. This process is essential to validate the target.

The article "Antiangiogenic Potential of Troxerutin and Chitosan Loaded Troxerutin on Chorioallantoic Membrane Model" was published in 2023. Journal: Biomed Res Int.

### 2.2. Molecular Docking

Molecular docking approach is employed to predict the binding interaction between the protein and ligand. Molecular docking was performed in glide ligand docking in the Schrodinger suite (Glide, Schrodinger, LLC, New York, NY, USA, 2021). The best compound was identified based on docking score. Glide extra precision scoring function is a novel scoring function to estimate the binding affinities. The top lead molecules were determined based on docking score.

### 2.3. Synthesis of Chitosan Nanoparticles Encapsulated with Troxerutin (Chi-Trox NPs)

Briefly, 100 mg of chitosan was weighed and added to the solution containing acetic acid and water (1 : 100 ratio). The solution was kept in magnetic stirrer at 200 rpm until chitosan was dissolved completely. To this solution, 0.1% Trox in ethanol was added and kept in magnetic stirrer at 200 rpm for overnight. To this, 10 ml sodium tri polyphosphate (STPP) was added with a final concentration of 0.35 g in 100 ml of distilled water. The solution was centrifuged at 10000 rpm for 10 minutes, and pellet was washed 3 times with distilled water. Finally Chi-Trox NPs were collected by dissolving the pellet in distilled water.

### 2.4. Characterization

A Malvern zeta sizer was used to quantify the particle size distributions of Trox and Chi-Trox NPs using dynamic light scattering (DLS). In order to evaluate the distribution of particle size of the drugs, 100 *μ*l of the Trox and Chi-Trox NPs were dissolved in 900 *μ*l of milliQ water. The surface morphology, size, and distribution of Trox and Chi-Trox nanoparticles were analyzed using scanning electron microscopy (SEM). Sonication was used to create a diluted sample that was well distributed. After that, the samples were dried and coated with a gold layer (sputter coating), visualized using a Qunta 200 SEM. Using Fourier transform infrared (FT-IR) spectroscopy with attenuated total reflection (ATR), the molecular vibrations of chitosan, Trox, and synthesized Chi-Trox NPs were examined. To study the spectra, a sufficient amount of material were deposited on the crystal surface, and peak values in the range of 500 cm^−1^ to 4000 cm^−1^ (Model BRUKER-ALPHA, Germany) were recorded using the OPUS program.

### 2.5. Drug Release Kinetic Assay

To study the drug release kinetics of synthesized Chi-Trox NPs, dialysis membrane method was used. The Trox and Chi-Trox NPs were suspended in distilled water. In 100 ml of phosphate buffer saline (PBS), the dialysis membrane was submerged. A magnetic stirrer was used to agitate the beaker at a speed of 250 rpm. An appropriate quantity of sample was removed from the beaker at specified time intervals (replaced with fresh PBS medium). UV-Vis spectrophotometer was used to analyze the samples at 480 nm.

The article "Antiangiogenic Potential of Troxerutin and Chitosan Loaded Troxerutin on Chorioallantoic Membrane Model" was published in 2023. Journal: Biomed Res Int.

### 2.6. Antiangiogenic Activity of Chi-Trox NPs on Chick Chorioallantoic Membrane (CAM)

During day 1, the eggs were wiped with ethanol, a small window (2 cm in diameter) was drilled on the egg shell, and 3 ml of albumin was removed using a 21 gauge needle. On day 3, under sterile conditions, a sterile disc was placed on top of the developing CAM. The discs were loaded with a 10 *μ*mol concentration of Trox and Chi-Trox NPs. The present work was grouped as follows: group I served as the control without any treatment. Group II received a 10 *μ*mol concentration of Trox. Group III received 10 *μ*mol concentrations of Chi-Trox NPs. After treatment with the appropriate drugs, the window on the egg was closed with sterile tape. The eggs were incubated at 37°C with a relative humidity (RH) of 50–60% until day 5. At the end of the 5th day, the egg windows were opened and the CAM membranes were photographed. The morphometric analysis of the Trox and Chi-Trox NPs was analyzed using the ImageJ software. The CAM membranes were collected and fixed in 10% formalin and stored at -20°C for further studies such as mRNA expression.

### 2.7. Anticancer Activity of Chi-Trox NPs on CAM

Freshly fertilized chicken eggs were incubated at a temperature of 37°C and a humidity of 50–60%. On the third day of embryo development, eggs were cleaned with ethanol, 3 ml of albumin was extracted through a tiny window on top of the CAM, and then eggs were parafilm-sealed. The egg window was opened on day 10, a filter disc was inserted inside, and 2 × 10^6^ HeLa cancer cells were transplanted into the disc. The window was then closed with parafilm. On day 14, egg windows were opened, 10 *μ*mol concentrations of Chi-Trox NPs and Trox were placed onto filter discs, and windows were sealed with parafilm. After three days of treatment, egg windows were opened, and tumor development on CAM tissues were collected and preserved in 10% formalin for further research.

### 2.8. Histopathological Examination of CAM

A 10% formalin fixative solution was flooded over the CAM area treated with Trox and Chi-Trox NPs. Using scissors and forceps, about 1 cm^2^ of membrane surrounding the treated area was carefully removed and dehydrated in various alcohol grades (50%, 70%, 90%, and absolute) followed by embedding in paraffin wax. A rotary microtome (Weswicox, Japan) was used to take vertical tissue sections (6 *μ*m). Before staining with hematoxylin and eosin, sections were treated with alcohol in progressive sequence of absolute, 90%, 70%, and 50% and cleaned with xylene. Qualitative assessment was conducted through the use of a light microscope at a magnification of 40x after mounting with digital picture exchange, and the pictures were captured using light microscope attached with a Nikon camera at 10x.

The article "Antiangiogenic Potential of Troxerutin and Chitosan Loaded Troxerutin on Chorioallantoic Membrane Model" was published in 2023. Journal: Biomed Res Int.

### 2.9. Immunohistochemistry Examination of CAM

A sterile container was used to collect the CAM membranes, and it was fixed in a 10% formalin solution. For 2 h, CAM paraffin slices (6 *μ*m) were incubated at 60°C on a heat plate. A xylene and ethanol solution was applied to dewaxed membrane sections followed by PBS wash. A heat plate was used for antigen retrieval at 37°C for 10 min, and 1% protease (Sigma-Aldrich, USA) was added. In order to reduce the amount of endogenous peroxidase activity in the sections, 0.3% hydrogen peroxide was used. The samples were then blocked with goat serum for 30 min prior to incubating overnight at 4°C with polyclonal anti-vimentin antibodies (1 : 500), anti-CD34 antibodies (1 : 500), and anti-CD44 antibodies (1 : 500). After this, the sections of membrane were incubated for 1 h at room temperature with goat secondary antibody (anti-mouse 1 : 500 (Dako, USA), followed by peroxidase-HRP conjugated at 1 : 500 (Dako). Diaminobenzidine/H_2_O_2_ substrate (Sigma-Aldrich, USA) was used to detect the immune reactivity. To counterstain the sections, 10% hematoxylin was applied and the sections were dehydrated and mounted in Pertex (Medite Medizintechnik, Germany).

### 2.10. Gene Expression Analysis by Real-Time PCR

TRIzol kit method was used to isolate the total RNA from the CAM. The isolated RNA was transcribed into cDNA using Takara kit method. All the primers sequences used in the current study were tabulated in Table 1. *β*-Actin was considered a reference gene. The RT-PCR assay was performed to amplify the gene of interest with SYBR green master mix (Takara, Japan). The following cycles were programmed during the amplification; initial denaturation at 95°C for 5 min followed by 40 cycles of 95°C for 30 s, 59–60°C for 30 s, and 72°C for 30 s.

### 2.11. Statistical Analysis

The analysis was carried out in triplicate, and all statistical data were presented as the mean ± standard deviation. GraphPad Prism version 9 was used to do one-way analysis of variance (ANOVA) and Duncan's multiple range tests to determine significant differences between mean values. The *p* < 0.05 values were deemed statistically significant.

The article "Antiangiogenic Potential of Troxerutin and Chitosan Loaded Troxerutin on Chorioallantoic Membrane Model" was published in 2023. Journal: Biomed Res Int.

## 3. Results and Discussion

### 3.1. Sequence Analysis

#### 3.1.1. Cluster of Differentiation 104 (CD104) Protein Modeling

Cluster of differentiation 104 (CD104) was retrieved from the Protein Data Bank (PDB ID 2YRZ). A three-dimensional structure of CD104 prepared in the protein preparation wizard embedded in the Schrodinger suite. In this process, we remove water molecules present in protein structure. Structure optimization includes optimization of hydrogen bond. Minimization restrained using OPLS_2005 force field. CD104 protein stereo chemical quality was analyzed using pro check in SAVES server. Ramachandran plot red color represents the most favored region is 84.4%. The yellow color region represent additional allowed region is 14.6%. The ramachandran plot for CD104 is shown in Figure 1.

*(1) Cluster of Differentiation 104 (CD104) Protein Modeling*.

#### 3.1.2. Vimentin Protein Modeling

Vimentin protein was retrieved from RCSB Protein Data Bank (PDB ID: 1GK4). The protein structure was imported using protein preparation wizard in the Schrodinger suite. Protein structure was preprocessed including assign bond order and replace hydrogen atoms, conversion of selenomethionines to methionines. Optimization of hydrogen bond was done; then, the structure was minimized using OPLS_2005 force field. The stereo chemical quality of a vimentin protein structure was analyzed using PROCHECK in SAVES server. Analysis was based on overall structure geometry as well as residue-by-residue geometry. Using PROCHECK, the Ramachandran plot was analyzed. The Ramachandran plot shows the most favored region is 96.7% and additional allowed region is 3.3%. The Ramachandran plot for vimentin protein was shown in Figure 2.

#### 3.1.3. Physicochemical Analysis

Physical and chemical properties of the protein were predicted in the expasy ProtParam tools. ProtParam tool predicts the number of amino acid, molecular weight, isoelectric point, total number of negatively charged residue, total number of positively charged residue, total number of atoms and their composition, aliphatic index, and grand average of hydropathicity (GRAVY). GRAVY value below zero indicates the hydrophilic nature of the protein. Hence, all the proteins (CD104 and vimentin) are hydrophilic in nature. Aliphatic index defined as the relative volume occupied by aliphatic amino acid side chain such as alanine, valine, and leucine. High aliphatic index (above 66.5) shows thermally stable over a wide temperature range. All these protein has a high aliphatic index, and these are protein thermally stable. Physicochemical properties of proteins were shown in Table 1.

The article "Antiangiogenic Potential of Troxerutin and Chitosan Loaded Troxerutin on Chorioallantoic Membrane Model" was published in 2023. Journal: Biomed Res Int.

### 3.2. Molecular Docking Studies

#### 3.2.1. Binding Poses of CD104 with Troxerutin

In glide docking protocol, troxerutin and cd104 were docked using glide ligand docking module in Schrodinger packages. Interacting residues between troxerutin and CD104 are Gln 55, Arg 89, Glu 103, and Glu101. Hydroxyl group of the ligand interacts with Gln 55 and forms hydrogen bonds with bond length of 2.17 Å. Arginine 89 interacts with ligand hydroxyl group forms hydrogen bond with distance 2.58 Å and pi-cation. Glutamic acid 103 interacts with ligand and forms 4 hydrogen bond interactions between the protein and ligand. Bond distance between the amino acid Glu 103 and ligand are 1.98 Å, 2.26 Å, 1.85 Å, and 2.31 Å. Interaction between protein and ligand molecules shows good binding affinity. Docking score was found to be -6.208 Kcal/Mol. Interactions between CD104 and troxerutin were shown in Figure 3.

#### 3.2.2. Binding Poses of Vimentin with Troxerutin

Vimentin protein was docked with troxerutin compound. Interacting residues are Glu192, Arg 196, and Thr 202. Glutamic acid residue at the position of 192 interacting with troxerutin forms 3 hydrogen bonds. Bond distance between protein and troxerutin is 1.73 Å, 1.73 Å, and 2.11 Å. Amino acid arginine residue at the position of 196 interacts with hydroxyl group of the troxerutin and form hydrogen bond with bond length of 2.44 Å. Thr 202 interacts with the ligand molecule forms hydrogen bond with distance of 2.05 Å. Docking score between vimentin and troxerutin was found to be -6.411. Interaction between troxerutin and vimentin protein was shown in Figure 4. Molecular docking interaction between proteins (CD104 and vimentin) and troxerutin was shown in Table 2.

### 3.3. Drug Encapsulation

Encapsulation and drug loading efficiency of chitosan NPs were 86.4 ± 0.12% and 13.2% ± 0.16%. Chitosan NPs show maximum encapsulation efficiency; after that, there is no change in encapsulation efficiency due to the polymer dispersion saturation.

### 3.4. Particle Size Measurement

Size and polydispersity index (PDI) are crucial assessments for the characterization of nanoparticles, since they affect crucial characteristics such as loading and the stability of the substance within nanoparticles. It is well known that the smaller the particle size, the larger the exposed surface area, which results in a quicker release of encapsulated therapeutics. Smaller particles also have a higher risk of aggregation during storage, making it crucial to design nanoparticles with a low PDI in order to maintain optimum stability through a more precise control of particle size. Notably, the repeatability of characteristics such as stability and release is closely related to a low PDI, as a large PDI indicates that the size distributions of the sample are not uniform. In the present study, the average particle size of Trox and Chi-Trox NPs were analyzed by the DLS as shown in Figure 5. The size of Trox and Chi-Trox NPs were found to be 896 d·nm and 692 d·nm, respectively, with a PDI of 0.885 and 0.355 (Figure 6). Results are in agreement with the previous studies reported by Luque-Alcaraz et al. [23], Ilk et al. [24], Li et al. [25] which were observed to have similar kind of results with chitosan encapsulated flavonoids.

The article "Antiangiogenic Potential of Troxerutin and Chitosan Loaded Troxerutin on Chorioallantoic Membrane Model" was published in 2023. Journal: Biomed Res Int.

### 3.5. FT-IR Analysis

FT-IR studies were carried out to confirm the similarity between Trox and Chi-Trox NPs (Figure 7). The FT-IR spectra of Trox showed peaks at 1058 cm^−1^ (C-O stretching), 1651 cm^−1^ (C=C stretching), 1752 cm^−1^ (C=O stretching), and 3324 cm^−1^ (O-H stretching). The FT-IR spectra of Chi-Trox showed peaks at 1020 cm^−1^ (C-N stretching), 1632 cm^−1^ (N-H stretching), 1740 cm^−1^ (C=O stretching), and 3333 cm^−1^ (O-H stretching). The presence of absorption band at 1223 cm^−1^ corresponding to P=O stretch indicates the interaction between phosphate groups of STPP and Chi-Trox NPs. No characteristic peaks of troxerutin were observed in the spectra, which may be indicative the presence of troxerutin was encapsulated with chitosan NPs, and this interaction was possibly occurred by hydrogen bonds or hydrophobic interactions. Similar kind of results were observed in previous studies reported by Hao et al. [26] and Kumar et al. [27].

### 3.6. SEM Analysis

Particle size and morphological studies of the Trox and synthesized Chi-Trox NPs were carried out using SEM (Figure 8). The microscopic image of Trox showed that the size was ranging 4 *μ*m with square shape. The microscopic images of Chi-Trox NPs were showed spherical shape morphology, with size ranging 500 nm. This happened because of high thermodynamic and shape stability of Chi-Trox NPs. Chi-Trox NPs have an agglomerated appearance due to ionic interactions between the drug, cross-linker, and polymer [28, 29].

### 3.7. Drug Release Kinetic Assay

The drug release profile of Chi-Trox NPs was analyzed, and it was compared with the native Trox (Figure 9). The Trox drug was released 6% in 3 hours whereas Chi-Trox NPs also released 6%. But after 9 hours, Chi-Trox NPs were released 31% in sustained manner and reached 85% after 18 hours whereas Trox released only 8% in 9 hours and 20% only in 18 hours. From the results, it was inferred that Chi-Trox NPs were releases more than native Trox. Similar types of results were observed in the previous studies in which chitosan encapsulated nanoparticles were released faster and sustained manner than the native forms [30–32].

The article "Antiangiogenic Potential of Troxerutin and Chitosan Loaded Troxerutin on Chorioallantoic Membrane Model" was published in 2023. Journal: Biomed Res Int.

### 3.8. Morphometric Analysis of CAM

The CAM assay provides *in vivo* evidence of angiogenesis. The CAM treated with Chi-Trox NPs (10 *μ*mol) showed significant decrease in the blood vessel density, total blood vessel network, total blood vessel branch points, and total blood vessel nets (*p* < 0.05) compared to the control and Trox (shown in Figure 8 and Table 3) The present study results were consistent with the previous reports [33, 34].

### 3.9. Histopathology Examination of CAM (Antiangiogenesis)

Using hematoxylin and eosin-stained sections of the CAM-treated area, we evaluated the morphological changes of the CAM to validate the antiangiogenic potential of Trox and Chi-Trox NPs (shown in Figure 10). The control CAM (without treatment) showed normal shape blood vessels and thick chorionic and allantoic epithelial layers. Large blood vessels were observed at the stromal area. In addition to this, congested small blood capillaries and protienaceous fluid was observed on surroundings of large blood vessels. The CAM treated with Trox showed irregular appearance of blood vessels at the thin chorionic and allantoic epithelial layer. Less number of large blood vessels were seen at stromal area compared the control. In addition to this, few small blood capillaries were seen around the large blood vessels. The CAM treated with Chi-Trox NPs showed comparatively thin chorionic and allantoic epithelial layer with diminished stromal area. Large blood vessels were not seen. Furthermore, very few small blood vessels were found compared to control and Trox indicates inhibition of sprouting. The results were inagreement with previously published articles [35, 36].

### 3.10. Immunohistochemistry Examination of CAM (Antiangiogenesis)

In the present study, we attempted to detect the expression levels of CD104 and vimentin on CAM using IHC (Figures 11 and 12). The results showed that CD104 was highly expressed in control CAM (without treatment) compared with and Trox and Chi-Trox NPs. The results of vimentin also showed high expression levels in the control group compared to Trox and Chi-Trox NPs. The results of this investigation indicated that Chi-Trox NPs could inhibit angiogenesis in CAM. These results were in agreement with the previously reported studies. van Beijnum et al. [37] reported the expression of vimentin antibody in CAM. The results revealed that vimentin expression in endothelial cells of CAM was reduced which resulted in the inhibition of angiogenesis. Nayak et al. [38] demonstrated the expression levels of vimentin in oral submucous fibrosis using IHC analysis. Chen and Wang [39] studied the prognostic value of vimentin in metastatic renal cell carcinoma (mRCC) using IHC. They revealed that expression of vimentin is associated with immunosuppression in mRCC and that the immunosuppressive status might be linked to the presence of programmed cell death ligand-1 (PDL-1) or programmed cell death protien-1 (PD-1) among those mRCCs. Liu et al. [40] demonstrated the expression of CD104 using IHC in prostate cancer, and results revealed that CD104 may play a key role as a biomarker in the prostate cancer.

The article "Antiangiogenic Potential of Troxerutin and Chitosan Loaded Troxerutin on Chorioallantoic Membrane Model" was published in 2023. Journal: Biomed Res Int.

### 3.11. mRNA Expression on CAM (Antiangiogenesis)

In the present investigation, the mRNA expression levels of MMP and FGF2 in tissues isolated from CAM in the control and treatment groups were analyzed by RT-PCR. Compared with control and Trox, the CAM treated with Chi-Trox NPs showed significant suppression in MMP and FGF2 mRNA expressions (*p* < 0.05) (Figures 13 and 14). Previously, few studies were reported on the mRNA expression profiling of MMP and FGF2 using RT-PCR. Hong et al. [41] demonstrated the mRNA expression of MMP-2 and MMP-9 in 3T3-L1 adipocyte cell lines. The results revealed that MMP-2 and MMP-9 levels were significantly decreased after treatment with quercetin compared with the control. Webb et al. [42] reported the mRNA expression of MMP-2 and MMP-9 in retinoblastoma cell lines. The results demonstrated that downregulation of MMP-2 and MMP-9 decreases the cell migration and angiogenesis. Bae et al. [43] demonstrated that the mRNA expression of MMP-2 and MMP-9 in HT1080 human fibro sarcoma cells was significantly downregulated after treatment with *L. tetragonum* plant extract. Wu et al. [44] demonstrated that FGF2 mRNA expression in HUVEC cell lines was significantly downregulated after treatment with formononetin.

### 3.12. Anticancer Activity on CAM

The cellular and morphological changes of CAM tumor sections were analyzed using macroscopic and histopathology (shown in Figures 15 and 16). The quantification of tumor size was evaluated and compared with the control. The results revealed that tumor size was significantly decreased upon treatment with Trox and Chi-Trox NPs (*p* < 0.01). The results demonstrated that control CAM (without treatment) showed a thick stratum, and more number of large blood vessels was observed between the allantoic and chorionic epithelial layer. Irregular appearance of blood vessels was observed at the subepithelium connective tissue. The CAM treated with Trox showed decrease in the blood cell formation with thin stratum. Few large blood vessels were seen compared to the control. The CAM treated with Chi-Trox NPs showed thin stratum, and large blood vessels were not seen compared to the control and Trox indicates the suppression of tumor. The immunohistochemical analysis showed high expression levels of CD44 compared to Trox and Chi-Trox NPs (Figure 17). The mRNA expression levels of FGF2 and MMP-9 on CAM treated with Chi-Trox NPs were significantly downregulated compared to the control and Trox (Figures 18 and 19). Similar type of results were observed in previous studies reported by Vu et al. [45] and Slekiene et al. [46].

The article "Antiangiogenic Potential of Troxerutin and Chitosan Loaded Troxerutin on Chorioallantoic Membrane Model" was published in 2023. Journal: Biomed Res Int.

## 4. Conclusion

The chitosan nanoparticles were successfully encapsulated with troxerutin and characterized by various analyses such as DLS, FT-IR, and SEM. The *in vitro* drug release kinetic assay confirmed that Chi-Trox NPs released sustained manner compared with Trox. The Chi-Trox NPs have more antiangiogenic potential than Trox by decreasing the blood vessel formation. Histopathology results showed decrease in the blood vessels formation supports the antiangiogenic ability. The immunohistochemical results showed low expression levels of CD104 and vimentin on endothelial cells (ECs) of CAM indicate inhibition of blood vessels. Furthermore, the mRNA expression levels of angiogenesis markers such as FGF2 and MMP were downregulated indicates its antiangiogenic activity. The anticancer activity results revealed suppression of tumor by inhibiting the blood vessel formation. The immunohistochemical results revealed low expression levels of CD44. Furthermore, the mRNA expression of FGF2 and MMP were downregulated indicates the anticancer activity. Altogether our findings suggest that Chi-Trox NPs could be a useful angiogenic inhibitor and can be more effectively used in future especially for the treatment of cancer.

## Figures and Tables

**Figure 1:** Ramachandran plot for cluster of differentiation 104 (CD104) protein.

**Figure 2:** Ramachandran plot for vimentin protein.

**Figure 3:** Interaction between troxerutin and CD104 protein.

**Figure 4:** Interaction between troxerutin and vimentin protein.

**Figure 5:** SEM results of (a) troxerutin and (b) Chi-Trox NPs.

**Figure 6:** DLS results of (a) troxerutin and (b) Chi-Trox NPs.

**Figure 7:** FT-IR results of (a) chitosan, (b) troxerutin, and (c) Chi-Trox NPs.

**Figure 8:** Chorioallantoic membrane *in ova* photographs showing vascular plexus after the incubation with control and treated groups (Trox and Trox-Chi NPs). (a) The photographs were taken after the treatment, incubation day-5. (b) Morphometric analysis of CAM treated with Trox and Chi-Trox NPs.

**Figure 9:** Drug release kinetic assay of Chi-Trox NPs.

**Figure 10:** Histological examinations of Chi-Trox NPs on CAM morphology: (a) control, (b) Trox, and (c) Chi-Trox NPs. lbv: large blood vessel; ae: allantoic epithelium; ce: chorionic epithelium.

The article "Antiangiogenic Potential of Troxerutin and Chitosan Loaded Troxerutin on Chorioallantoic Membrane Model" was published in 2023. Journal: Biomed Res Int.

**Figure 11:** Immunohistostaining of CD104 in chick embryo chorioallantoic membranes (CAM): (a) control, (b) Trox, and (c) Chi-Trox.

**Figure 12:** Immunohistostaining of vimentin in chick embryo chorioallantoic membranes (CAM): (a) control, (b) Trox, and (c) Chi-Trox. Red arrow shows expression of vimentin.

**Figure 13:** Effects of Trox and Chi-Trox NPs on the expression of FGF2 in chick chorioallantoic membrane. Comparison made between control and Trox, control and Chi-Trox NPs. Trox: troxerutin; Chi-Trox NPs: chitosan nanoparticles encapsulated with troxerutin; SD: standard deviation. The statistical analysis was done by using ANOVA and Tukey's post hoc test. ^∗^significant difference compared with control (*p* < 0.05); ^∗∗^significant difference compared with the control (*p* < 0.01); ^∗∗∗^significant difference compared with the control (*p* < 0.001); and ^∗∗∗∗^significant difference compared with the control (*p* < 0.0001).

**Figure 14:** Effects of Trox and Chi-Trox NPs on the expression of MMP in chick chorioallantoic membrane. Comparison made between control and Trox and control and Chi-Trox NPs; Trox: troxerutin; Chi-Trox NPs: chitosan nanoparticles encapsulated with troxerutin; SD: standard deviation. The statistical analysis was done by using ANOVA and Tukey's post hoc test. ^∗^Significant difference compared with the control (*p* < 0.05); ^∗∗^significant difference compared with the control (*p* < 0.01); ^∗∗∗^significant difference compared with the control (*p* < 0.001); ^∗∗∗∗^significant difference compared with the control (*p* < 0.0001).

**Figure 15:** (a) Inhibition of growth in HeLA cells in the CAM by Trox and Chi-Trox NPs. (b) Quantification of A498 cell tumor size after treatment with Trox and Chi-Trox NPs using box plot.

**Figure 16:** Histological examinations of Chi-Trox NPs on CAM morphology: (a) control, (b) Trox, and (c) Chi-Trox NPs. lbv: large blood vessel; ae: allantoic epithelium; ce: chorionic epithelium.

**Figure 17:** Immunohistostaining of CD44 in chick embryo chorioallantoic membranes (CAM): (a) control, (b) Trox, and (c) Chi-Trox.

**Figure 18:** Anticancer effects of Trox and Chi-Trox NPs on the expression of FGF2 in chick chorioallantoic membrane. Comparison made between control and Trox and control and Chi-Trox NPs; Trox: troxerutin; Chi-Trox NPs: chitosan nanoparticles encapsulated with troxerutin; SD: standard deviation. The statistical analysis was done by using ANOVA and Tukey's post hoc test. ^∗^Significant difference compared with the control (*p* < 0.05); ^∗∗^significant difference compared with the control (*p* < 0.01); ^∗∗∗^significant difference compared with the control (*p* < 0.001); ^∗∗∗∗^significant difference compared with the control (*p* < 0.0001).

The article "Antiangiogenic Potential of Troxerutin and Chitosan Loaded Troxerutin on Chorioallantoic Membrane Model" was published in 2023. Journal: Biomed Res Int.

**Figure 19:** Anticancer effects of Trox and Chi-Trox NPs on the expression of MMP in chick chorioallantoic membrane. Comparison made between control and Trox and control and Chi-Trox NPs. Trox: troxerutin; Chi-Trox NPs: chitosan nanoparticles encapsulated with troxerutin; SD: standard deviation. The statistical analysis was done by using ANOVA and Tukey's post hoc test. ^∗^Significant difference compared with the control (*p* < 0.05); ^∗∗^significant difference compared with the control (*p* < 0.01); ^∗∗∗^significant difference compared with the control (*p* < 0.001); ^∗∗∗∗^significant difference compared with the control (*p* < 0.0001).

**Table 1:** Physiochemical properties of CD104 and vimentin.

Properties	CD104	Vimentin
Number of amino acids	118	84
Molecular weight (Da)	12	10
Theoretical pI	5.89	4.54
Total number of negatively charged residue (Asp+Glu)	12	22
Total number of positively charged residue (Arg+Lys)	10	16
Number of atoms	1774	1461
Aliphatic index	76.69	91.86
Grand average of hydropathicity (GRAVY)	-0.520	-1.047

**Table 2:** Docking analysis of CD104 and vimentin with troxerutin.

S. no.	Docking complexes	Docking score (Kcal/Mol)	Interacting residues with distance
1.	CD104_Toxerutin	-6.208	Gln_55 (2.17 Å), Arg_89 (2.58 Å), Arg_100 (2.87 Å), Glu 101 (1.84 Å) and 103 (1.98 Å, 2.26 Å, 1.85 Å, and 2.31 Å)
2.	Vimentin_Troxerutin	-6.411	Glu_192 (1.73 Å, 1.73 Å, and 2.11 Å), Arg _196 (2.44 Å), Thr_202 (2.05 Å)

**Table 3:** Morphometric analysis of Trox and Chi-Trox NPs in chick embryo chorioallantoic membrane (CAM) using ImageJ software.

Group	Blood vessel density (mean ± SD)	Total vessel network (mean ± SD)	Total branching points (mean ± SD)	Total nets (*mean* ± *SD*)
Control	26.66 ± 1.52	34648 ± 818.51	94 ± 3.51	31 ± 2
Trox 10 *μ*mol	20.46 ± 0.55^a^∗^^	30223 ± 1664.1^a^∗^^	62 ± 1.52^a^∗^^	24 ± 2^a^∗^^
Chi-Trox 10 *μ*mol	14.76 ± 1.72^b∗c∗^	18898 ± 989^b∗c∗^	31 ± 2^b∗c∗^	11.66 ± 1.52^b∗c∗^

Comparison made between control and Trox, Control and Chi-Trox NPs, and Trox and Chi-Trox NPs. SD: standard deviation; statistical analysis was done by using student *t*-test; ^a^^∗^significant difference of Trox compared with the control (*p* < 0.05), ^b^^∗^significant difference of Chi-Trox NPs compared with the control (*p* < 0.05); and ^c^^∗^significant difference of Chi-Trox NPs compared with Trox (*p* < 0.05).

## Data Availability

All data used to support the fndings of this study are available from the corresponding author upon request.

The article "Antiangiogenic Potential of Troxerutin and Chitosan Loaded Troxerutin on Chorioallantoic Membrane Model" was published in 2023. Journal: Biomed Res Int.

## Abbreviations

Trox: Troxerutin
Chi-Trox NPs: Chitosan encapsulated troxerutin nanoparticles
CAM: Chick chorioallantoic membrane
IHC: Immunohistochemistry
VEGF: Vascular endothelial growth factor
MMP: Matrix metalloproteinase
FGF2: Fibroblast growth factor-2
DLS: Dynamic light scattering
SEM: Scanning electron microscope
FT-IR: Fourier-transform infrared.

## References

[1] Eelen G., Treps L., Li X., Carmeliet P. (2020). Basic and therapeutic aspects of angiogenesis updated. *Circulation Research*.

[2] O'Reilly M. S., Boehm T., Shing Y. (1997). Endostatin: an endogenous inhibitor of angiogenesis and tumor growth. *Cell*.

[3] Curry J. M., Eubank T. D., Roberts R. D. (2008). M-CSF signals through the MAPK/ERK pathway via Sp1 to induce VEGF production and induces angiogenesis in vivo. *PLoS One*.

[4] Abdolmaleki Z., Arab H. A., Amanpour S., Muhammadnejad S. (2016). Anti-angiogenic effects of ethanolic extract of *Artemisia sieberi* compared to its active substance, artemisinin. *Revista Brasileira de Farmacognosia*.

[5] Panche A. N., Diwan A. D., Chandra S. R. (2016). Flavonoids: an overview. *Journal of Nutritional Science*.

[6] Fu Y., Liu W., Soladoye O. P. (2021). Towards innovative food processing of flavonoid compounds: insights into stability and bioactivity. *LWT*.

[7] Kumar S., Pandey A. K. (2013). Chemistry and biological activities of flavonoids: an overview. *The Scientific World Journal*.

[8] Ahmadi Z., Mohammadinejad R., Roomiani S., Afshar E. G., Ashrafizadeh M. (2021). Biological and therapeutic effects of troxerutin: molecular signaling pathways come into view. *Journal of Pharmaco Puncture*.

[9] Shan Q., Zhuang J., Zheng G. (2017). Troxerutin reduces kidney damage against BDE-47-induced apoptosis via inhibiting NOX2 activity and increasing Nrf2 activity. *Oxidative Medicine and Cellular Longevity*.

[10] Lazer L. M., Sadhasivam B., Palaniyandi K. (2018). Chitosan-based nano-formulation enhances the anticancer efficacy of hesperetin. *International Journal of Biological Macromolecules*.

[11] Narayan S., Jana S., Jana S. (2019). Chitosan-Based Nanoformulation as Carriers of Small Molecules for Tissue Regeneration. *Functional Chitosan*.

[12] Vedakumari W. S., Ayaz N., Karthick A. S., Senthil R., Sastry T. P. (2017). Quercetin impregnated chitosan–fibrin composite scaffolds as potential wound dressing materials—fabrication, characterization and in vivo analysis. *European Journal of Pharmaceutical Sciences*.

[13] Anitha A., Deepagan V. G., Rani V. D., Menon D., Nair S. V., Jayakumar R. (2011). Preparation, characterization, *in vitro* drug release and biological studies of curcumin loaded dextran sulphate -chitosan nanoparticles. *Carbohydrate Polymers*.

The article "Antiangiogenic Potential of Troxerutin and Chitosan Loaded Troxerutin on Chorioallantoic Membrane Model" was published in 2023. Journal: Biomed Res Int.

[14] Bilia A. R., Guccione C., Isacchi B., Righeschi C., Firenzuoli F., Bergonzi M. C. (2014). Essential oils loaded in nanosystems: a developing strategy for a successful therapeutic approach. *Evidence-based Complementary and Alternative Medicine*.

[15] Raza Z. A., Khalil S., Ayub A., Banat I. M. (2020). Recent developments in chitosan encapsulation of various active ingredients for multifunctional applications. *Carbohydrate Research*.

[16] Victorelli F. D., de Oliveira Cardoso V. M., Ferreira N. N. (2020). Chick embryo chorioallantoic membrane as a suitable *in vivo* model to evaluate drug delivery systems for cancer treatment: A review. *European Journal of Pharmaceutics and Biopharmaceutics*.

[17] Nowak-Sliwinska P., Segura T., Iruela-Arispe M. L. (2014). The chicken chorioallantoic membrane model in biology, medicine and bioengineering. *Angiogenesis*.

[18] Altschul S. F., Gish W., Miller W., Myers E. W., Lipman D. J. (1990). *Basic local alignment search tool*. *Molecular Biology*.

[19] Gasteiger E., Hoogland C., Gattiker A., Walker J. M. (2005). Protein Identification and Analysis Tools on the ExPASy Server. *The Proteomics Protocols Handbook. Springer Protocols Handbooks*.

[20] Zheng W., Wuyun Q., Zhou X., Li Y., Freddolino P., Zhang Y. (2022). LOMETS3: integrating deep learning and profile alignment for advanced protein template recognition and function annotation. *Nucleic Acids Research*.

[21] Ko J., Park H., Heo L., Seok C. (2012). GalaxyWEB server for protein structure prediction and refinement. *Nucleic Acids Research*.

[22] Laskowski R. A., MacArthur M. W., Moss D. S., Thornton J. M. (1993). PROCHECK: a program to check the stereochemical quality of protein structures. *Journal of Applied Crystallography*.

[23] Luque-Alcaraz A. G., Lizardi J., Goycoolea F. M. (2012). Characterization and antiproliferative activity of nobiletin-loaded chitosan nanoparticles. *Journal of Nanomaterials*.

[24] Ilk S., Saglam N., Özgen M. (2017). Kaempferol loaded lecithin/chitosan nanoparticles: preparation, characterization, and their potential applications as a sustainable antifungal agent. *Artificial Cells, Nanomedicine, and Biotechnology*.

[25] Li F., Shi Y., Liang J., Zhao L. (2019). Curcumin-loaded chitosan nanoparticles promote diabetic wound healing via attenuating inflammation in a diabetic rat model. *Journal of Biomaterials Applications*.

[26] Hao J., Guo B., Yu S. (2017). Encapsulation of the flavonoid quercetin with chitosan-coated nano-liposomes. *LWT- Food Science and Technology*.

[27] Kumar S. P., Birundha K., Kaveri K., Devi K. R. (2015). Antioxidant studies of chitosan nanoparticles containing naringenin and their cytotoxicity effects in lung cancer cells. *International Journal of Biological Macromolecules*.

The article "Antiangiogenic Potential of Troxerutin and Chitosan Loaded Troxerutin on Chorioallantoic Membrane Model" was published in 2023. Journal: Biomed Res Int.

[28] Arulmozhi V., Pandian K., Mirunalini S. (2013). Ellagic acid encapsulated chitosan nanoparticles for drug delivery system in human oral cancer cell line (KB). *Colloids and Surfaces B: Biointerfaces*.

[29] Yusefi M., Chan H. Y., Teow S. Y. (2021). 5-fluorouracil encapsulated chitosan-cellulose fiber bionanocomposites: synthesis, characterization and in vitro analysis towards colorectal cancer cells. *Nano Materials*.

[30] Das R. K., Kasoju N., Bora U. (2010). Encapsulation of curcumin in alginate-chitosan-pluronic composite nanoparticles for delivery to cancer cells. *Nanomedicine: Nanotechnology, Biology and Medicine*.

[31] Onyebuchi C., Kavaz D. (2019). Chitosan and N, N, N-trimethyl chitosan nanoparticle encapsulation of *Ocimum Gratissimum* essential oil: optimised synthesis, in vitro release and bioactivity. *International Journal of Nanomedicine*.

[32] Nair R. S., Morris A., Billa N., Leong C. O. (2019). An evaluation of curcumin-encapsulated chitosan nanoparticles for transdermal delivery. *AAPS PharmSciTech*.

[33] Rahmani F., Karimi E., Oskoueian E. (2020). Synthesis and characterisation of chitosan-encapsulated genistein: its anti-proliferative and anti-angiogenic activities. *Journal of Microencapsulation*.

[34] Sanatkar R., Rahimi Kalateh Shah Mohammad G., Karimi E., Oskoueian E., Hendra R. (2022). Evaluation of daidzein-loaded chitosan microcapsules for the colon cancer drug delivery: synthesis, characterization and release behaviour. *Polymer Bulletin*.

[35] Manjunathan R., Ragunathan M. (2015). In ovo administration of human recombinant leptin shows dose dependent angiogenic effect on chicken chorioallantoic membrane. *Biological Research*.

[36] Bessa G., Melo-Reis P. R., Araújo L. A. (2015). Angiogenic activity of latex from Euphorbia tirucalliLinnaeus 1753 (Plantae, Euphorbiaceae). *Brazilian Journal of Biology*.

[37] van Beijnum J. R., Huijbers E. J., van Loon K. (2022). Extracellular vimentin mimics VEGF and is a target for anti-angiogenic immunotherapy. *Nature Communications*.

[38] Nayak M. T., Singh A., Desai R. S., Vanaki S. S. (2013). Immunohistochemical analysis of vimentin in oral submucous fibrosis. *Journal of Cancer Epidemiology*.

[39] Chen X., Wang H. (2020). Prognostic value of vimentin is associated with immunosuppression in metastatic renal cell carcinoma. *Frontiers in Oncology*.

[40] Liu A. Y., Roudier M. P., True L. D. (2004). Heterogeneity in primary and metastatic prostate cancer as defined by cell surface CD profile. *The American Journal of Pathology*.

[41] Hong S. Y., Ha A. W., Kim W. (2021). Effects of quercetin on cell differentiation and adipogenesis in 3T3-L1 adipocytes. *Nutrition Research and Practice*.

The article "Antiangiogenic Potential of Troxerutin and Chitosan Loaded Troxerutin on Chorioallantoic Membrane Model" was published in 2023. Journal: Biomed Res Int.

[42] Webb A. H., Gao B. T., Goldsmith Z. K. (2017). Inhibition of MMP-2 and MMP-9 decreases cellular migration, and angiogenesis in in vitro models of retinoblastoma. *BMC Cancer*.

[43] Bae M. J., Karadeniz F., Oh J. H. (2017). MMP-Inhibitory Effects of Flavonoid Glycosides from Edible Medicinal Halophyte *Limonium tetragonum*. *Evidence-based Complementary and Alternative Medicine*.

[44] Wu X. Y., Xu H., Wu Z. F. (2015). Formononetin, a novel FGFR2 inhibitor, potently inhibits angiogenesis and tumor growth in preclinical models. *Oncotarget*.

[45] Vu B. T., Shahin S. A., Croissant J. (2018). Chick chorioallantoic membrane assay as an *in vivo* model to study the effect of nanoparticle-based anticancer drugs in ovarian cancer. *Scientific Reports*.

[46] Slekiene L., Stakisaitis D., Balnyte I., Valanciute A. (2018). Sodium valproate inhibits small cell lung cancer tumor growth on the chicken embryo chorioallantoic membrane and reduces the p53 and EZH2 expression. *Dose-Response*.

